# A Comparison between Three-Dimensional Visualization Guided Hepatectomy and Ultrasonography Guided Radiofrequency Ablation in the Treatment of Small Hepatocellular Carcinoma within the Milan Criteria

**DOI:** 10.1155/2016/8931732

**Published:** 2016-05-12

**Authors:** Tian-pei Guan, Chi-hua Fang, Jian Yang, Nan Xiang, Qing-shan Chen, Shi-zhen Zhong

**Affiliations:** ^1^Department of Hepatobiliary Surgery, Zhujiang Hospital, Southern Medical University, Guangzhou, Guangdong 510282, China; ^2^The Clinical Anatomy Institute, Southern Medical University, Guangzhou, Guangdong 510515, China

## Abstract

*Background*. Treatment selection for small hepatocellular carcinoma (sHCC) is controversial. We aimed to compare the outcomes of medical imaging three-dimensional visualization system (MI-3DVS) guided surgical resection (SR) and ultrasonography guided radiofrequency ablation (RFA) for sHCC.* Methods*. In total, 194 patients who underwent SR or RFA in our hospital between January 2006 and May 2010 were retrospectively enrolled. Overall survival (OS), recurrence-free survival (RFS), and postoperative complications were compared. Cox regression was used to estimate the benefits of MI-3DVS-guided SR on OS and RFS.* Results*. Ninety-two patients underwent SR and 102 underwent RFA. The SR group experienced more complications (41.3% versus 19.6%) and longer hospital stay (18.04 ± 7.11 versus 13.06 ± 5.59) (both *p* < 0.05). The 1-, 2-, 3-, 4-, and 5-year OS was 96.7%, 95.7%, 93.5%, 83.5%, and 61.1% in the SR group and 95.0%, 88.1%, 72.7%, 56.9%, and 39.5% in the RFA group. Corresponding RFS was 95.7%, 94.6%, 84.7%, 59.8%, and 40.2% in SR group and 91.2%, 80.3%, 60.5%, 32.3%, and 22.3% in RFA group. The 5-year OS and RFS were higher in SR group (both *p* < 0.001). Interestingly, there was no significance in OS and RFS among subgroups aged >60 years. Independent predictors of OS and RFS, respectively, were intervention (HR, 2.769 and 1.933), tumor number (HR, 5.128 and 3.903), and serum alpha-fetoprotein (AFP) (HR, 1.871 and 1.474) (all *p* < 0.05).* Conclusions*. MI-3DVS based hepatectomy should be considered primary treatment while RFA can be treated as alternative therapy for older patients. Intervention, tumor number, and AFP are independent predictors for both survival and recurrence.

## 1. Introduction

Hepatocellular carcinoma (HCC) is the second leading cause of cancer associated death worldwide [1]. Although Asian countries account for more than 70% of HCC cases [2], rising trends in morbidity and mortality in Western countries have been reported [1, 3]. Surgical resection (SR), transplantation, and radiofrequency ablation (RFA) are recommended as curative methods for patients at the early stage in the Barcelona Clinic Liver Cancer system [4] and those who meet the Milan criteria [2, 5]. RFA is characterized by high cost-effectiveness and minimal invasiveness while SR is considered a high-risk intervention. To reduce the performance-related risks, several surgery planning software systems have been developed [6–8]. To the best of our knowledge, the long-term outcomes of these technique based SR have not been analyzed. This study aimed to compare the outcomes of medical imaging three-dimensional visualization system (MI-3DVS, patented by the authors; software copyright number 2008SR18798) based SR and RFA in patients with sHCC who met the Milan criteria and to identify the predictors of survival and recurrence.

## 2. Material and Methods

### 2.1. Patients and Definitions

HCC patients who underwent MI-3DVS based SR or ultrasonography guided RFA as the initial treatment in Zhujiang Hospital between January 2006 and May 2010 and met the eligibility criteria were retrospectively enrolled. The diagnosis of HCC was mainly based on typical features such as arterial hypervascularity and wash out in the early or delayed venous phase on 4-phase contrast-enhanced computed tomography (CT) or dynamic contrast-enhanced magnetic resonance imaging (MRI) [4]. Ultrasonography or CT-guided biopsy was performed when the diagnosis was dubious according to the practice guidelines [4, 9]. Tumor number and diameter were calculated based on the MI-3DVS and/or CT/MRI findings as previously reported [7]. The severity of postoperative complications was estimated according to the Clavien-Dindo Classification system [10]. Demographic and clinical data were retrieved from the hospital's data center. Tumor recurrence was defined as the emergence of lesions within the liver parenchyma or outside the liver at least 4 weeks after treatment.

Eligibility criteria were as follows: (1) meeting the Milan criteria (single HCC ≤ 5 cm or no more than 3 lesions with the largest nodule ≤ 3 cm in diameter); (2) no evidence of extrahepatic metastasis or vascular invasion or extensive lymph node metastasis; (3) Child-Pugh liver function class A or B; (4) no history of encephalopathy, refractory ascites, or variceal bleeding; and (5) no history of anticancer treatment.

### 2.2. Follow-Up

The main endpoints of this study were cumulative OS, recurrence-free survival (RFS), and postoperative complications. The patients were routinely required to revisit our hospital for follow-up 4 weeks after treatment. Then, serum alpha-fetoprotein (AFP) levels were measured and ultrasonography was performed every 2-3 months for 2 years and then every 6 months for up to 5 years. When intrahepatic recurrence was equivocal, MRI or contrast-enhanced CT was performed. In patients with suspected extrahepatic recurrence, chest CT or positron emission tomography was performed. Once recurrence was confirmed, hepatectomy, RFA, percutaneous ethanol injection (PEI), transcatheter hepatic arterial chemoembolization (TACE), or treatment with sorafenib was recommended.

### 2.3. Three-Dimensional Visualization and Surgery Planning

The process of three-dimensional (3D) reconstruction and the requirements of the CT dataset by the system have been described previously [7, 11]. The enhanced thin CT slices (2 mm) were automatically registered by the software. Based on the CT data, a 3D model and corresponding individual Couinaud's anatomic segmentation of the liver could be successfully reconstructed by MI-3DVS according to the distribution area of the hepatic vein and the shape of the portal vein. After that, the 3D liver models were derived as a Standard Template Library file and imported to the Free Form Modeling System (SensAble Technologies, Inc., TextureKiln, USA) to visualize the regions of interest such as the hepatic artery blood supply, location of the HCC, and vascular variations. The total volume and remnant volume of the liver after tumor resection as well as the percentage of the remnant liver were automatically calculated by the measurement tool attached to the Free Form Modeling System. Then, an appropriate strategy was decided according to these parameters. While the operation was performed, the reconstructed models as well as the planed hepatectomy were displayed on a portable computer in the operating room to provide indirect guidance.

### 2.4. Radiofrequency Ablation

RFA was carried out using the Radionics Cool-Tip RF Ablation System (Radionics, Burlington, VT, USA) under ultrasonography guidance (ACUSON SEQUOIA*™* 512 Ultrasound System, Siemens, Berlin, Germany). The procedure was performed with the patient under local, intravenous, or spinal anesthesia, based on their preference. The placement of the ablation needle was achieved under ultrasonography guidance. After appropriate placement, RFA was activated from 10 W to 120 W with an increase of 10 W per minute. Then, RFA was sustained until a total ablative area of 0.5–1.0 cm over the tumor margin in ultrasonography images or an obvious impedance increase of ≥10 Ω appeared.

### 2.5. Statistical Analysis

The sample size was calculated with a 5-year overall survival (OS) rate equal to 60% in the SR group and 40% in the RFA group using Empower Stats software (X&Y Solutions Inc., Boston, USA). The type-I error and power were set at 0.05 and 0.90 for a 2-sided log-rank test. Therefore, at least 75 patients were needed in each group, with an estimated lost to follow-up rate of 20%.

The Student *t*-test and *χ* ^2^ tests were employed for continuous data and categorical data. The Mann-Whitney *U* test was used for the ranked data. The Kaplan-Meier method with the log-rank test was used to generate survival functions and estimate the significance between the groups. Cumulative survival rates were estimated with survival tables using the log-rank test. Bivariate and partial correlation analyses were performed to identify factors associated with OS and RFS. The factors identified by correlation analysis were analyzed by both univariate and multivariate analyses using Cox proportional hazards regression models to identify the risk factors associated with survival and recurrence. Statistical analyses were performed using the SPSS 13.0 for Windows (SPSS Inc., IL, USA). A *p* value <0.05 was considered statistically significant.

### 2.6. Ethics Statement

This study was approved by the Ethics Committee of Zhujiang Hospital, Southern Medical University (Number 2014-GDYK-007). Although written informed consent was not required because of the retrospective study design, the patients were informed that their data would be used for scientific purpose when they were hospitalized.

## 3. Results

### 3.1. Patient Characteristics

A total of 194 patients who met the eligibility criteria were enrolled in the present study and analyzed. Among these subjects, 92 (47.4%) underwent SR and 102 (52.6%) underwent RFA. Of the patients, 75 in the SR group and 90 in the RFA group were men. The mean age was 52.48 ± 8.36 years and 54.02 ± 7.66 years in the SR and RFA groups, respectively. 3D models were successfully reconstructed the patients in SR group (Figure 1). The diameter of the lesions in the SR and RFA groups was 3.14 ± 1.06 cm and 3.17 ± 0.91 cm, respectively. In addition, the number of patients with 1, 2, or 3 tumors, respectively, was 67, 18, and 7 in the SR group and 68, 22, and 12 in the RFA group. There were no significant differences in sex, age distribution, tumor number, tumor diameter, liver function, hepatitis virus infection, alcoholism, cirrhosis, and results of blood biochemical tests between the two groups (all *p* > 0.05) (Table 1).

### 3.2. Postoperative Complications and Clavien-Dindo Classification

Patients who underwent liver resection experienced longer hospital stay than those who received RFA (18.04 ± 7.11 versus 13.06 ± 5.59 days, *p* < 0.001). The incidence of procedure-related complications was higher in the SR group than in the RFA group (38/92 versus 20/102, *p* = 0.001). Major complications in the SR group were hydrothorax (4 cases), ascites (7), bile leakage (2), postoperative hemorrhage (1), fever ≥38.5°C for at least 3 days (5), and severe pain (23). Major complications in the RFA group were hydrothorax (2 cases), ascites (2), postoperative hemorrhage (1), hepatic failure (1), massive necrosis (1), pneumothorax (3), fever ≥38.5°C for at least 3 days (2), and severe pain (8). Additionally, the rate of moderate-severe complications (Clavien-Dindo class ≥ grade 2) in the SR group was significantly higher than in the RFA group (19/92 versus 4/102, *p* < 0.001). Further details regarding postoperative complications are presented in Table 2.

### 3.3. Overall Survival and Recurrence-Free Survival

The median (quartile range) follow-up periods in the SR and RFA groups were 60 (50–60) months and 48.5 (28–60) months, respectively. During this period, 23 patients (9 in the SR group and 14 in the RFA group) were lost to follow-up, and 94 patients (35 in the SR group and 59 in the RFA group) died of HCC-related disease. The major causes of death were tumor progression, liver failure, massive hemorrhage, and hepatic encephalopathy. Three patients died because of other reasons (1 for unknown reason in the SR group; 1 suicide and 1 traffic accident in the RFA group). There were no treatment-related deaths in either group during the 3 months after treatment. In total, 124 patients experienced recurrence (52 in the SR group and 72 in the RFA group). Treatments for recurrence are summarized in Table 3.

The 1-, 2-, 3-, 4-, and 5-year OS rates were, respectively, 96.7%, 95.7%, 93.5%, 83.5%, and 61.1% in the SR group and 95.0%, 88.1%, 72.7%, 56.9%, and 39.5% in the RFA group. The corresponding RFS rates were 95.7%, 94.6%, 84.7%, 59.8%, and 40.2% in the SR group and 91.2%, 80.3%, 60.5%, 32.3%, and 22.3% in the RFA group. Both OS and RFS were significantly higher in patients who underwent hepatectomy than in those who received RFA (Figure 2).

Additionally, in the SR group, both OS and RFS were higher among subgroups of patients with solitary HCC ≤ 3 cm, multifocal HCC, solitary HCC > 3 cm, serum AFP level ≥ 400 *μ*g/L, serum AFP level < 400 *μ*g/L, Child-Pugh class A, Child-Pugh class B, and younger patients (aged ≤ 60 years). However, no significant differences in RFS were found in patients with multiple nodules and Child-Pugh class B and in older patients (aged > 60 years) (Table 4).

### 3.4. Prognostic Indicators for Survival and Recurrence

The factors associated with OS in correlation analysis (disregarding the strength of the association) were intervention, tumor number, tumor diameter, Child-Pugh class, cirrhosis, serum AFP, and tumor recurrence. The factors associated with RFS were intervention, tumor number, tumor diameter, Child-Pugh class, and serum AFP, respectively (Table 5). These variables were analyzed by using the Cox proportional hazards model to identify the independent predictors of survival and tumor recurrence. By univariate analysis, the factors associated with OS were intervention, tumor number, serum AFP, Child-Pugh class, and tumor recurrence. However, by multivariate analysis, tumor diameter was associated with OS while tumor recurrence, Child-Pugh class, and tumor recurrence were not. The corresponding hazard ratios (HRs) were 2.769 (95% confidence interval (CI): 1.789–4.286, *p* < 0.001) for intervention, 2.166 (95% CI: 1.656–2.835, *p* < 0.001) for tumor diameter (cm), 5.128 (95% CI: 3.548–7.413, *p* < 0.001) for tumor number, and 1.871 (95% CI: 1.229–2.847, *p* = 0.003) for serum AFP.

By univariate analysis, the factors associated with RFS were intervention, tumor number, serum AFP, Child-Pugh class, and tumor recurrence. However, by multivariate analysis, Child-Pugh class was not associated with RFS while tumor diameter was. The corresponding HRs for intervention, tumor number, tumor diameter, and serum AFP were 1.933 (95% CI: 1.340–1.789, *p* < 0.001), 3.903 (95% CI: 2.819–5.404, *p* < 0.001), 1.411 (95% CI: 1.132–1.759, *p* = 0.002), and 1.474 (95% CI: 1.023–2.126, *p* = 0.038), respectively. Further details are provided in Tables 6 and 7.

## 4. Discussion

HCC is the sixth most common malignancy and the second leading cause of cancer associated death globally [1, 12]. Liver transplantation, RFA, and liver resection are recommended curative methods for HCC by the European Association for the Study of the Liver, European Organization for Research and Treatment of Cancer, and the American Association for the Study of Liver Diseases guidelines [4, 9]. However, SR remains to be the preferred treatment for HCC because of donor scarcity, especially in Asian countries [2, 7]. Tumor number and size and underlying disease as well as venous and/or artery variations play an important role in treatment decisions, especially in patients with combined cirrhosis [13], for whom more remnant volume should be reserved to ensure the safety of the surgery. Severe surgery-related complications such as liver dysfunction and bile leakage are closely associated with improper management of the intrahepatic vessels during the operation [14]. Comprehensive understanding of the tumor characteristics and adjacent structures is critical for successful patient management [11, 15, 16]. Developments in computer science and its integration with medical imaging technology offer a novel opportunity to reduce these adverse events by visualizing the intrahepatic vessels and optimizing resection schemes on individual 3D models. The application of MI-3DVS in observing the origin, bifurcations, and anatomical variations of blood vessels and the relationship between the tumor and crucial surrounding structures have been described previously [17–20]. This technology plays an important role in volumetric analysis and characterizing the anatomical features of hepatolithiasis, liver cancer, and pancreatic disease [7, 8, 17, 21]. In other words, major drawbacks of conventional hepatectomy, such as compromised liver function and high incidence of complications could be overcome or at least minimized through adequate preservation of liver parenchyma and comprehensive preoperative evaluation. The present study showed that sHCC patients who meet the Milan criteria could benefit more from MI-3DVS-guided SR than RFA in terms of better survival and lower recurrence rate.

The results of our study showed that patients who underwent SR experienced longer hospital stay than those who received RFA. Consistent with previous studies [22–25], the incidence of procedure-related complications as well as the rate of serve complications in the SR group was significantly higher than that in the RFA group. Interestingly, the incidence of procedure-related severe adverse events (grade III-IV) in the present study, such as bile leakage, postoperative hemorrhage hydrothorax, and hepatic failure, was much lower than that reported in patients who underwent conventional hepatectomy for HCC in a randomized prospective clinical trial (3/92 versus 13/100, resp.) [26]. This difference may be explained by the fact that the MI-3DVS allows preoperative planning. The 3D model of the MI-3DVS facilitates the localization of lesions and identification of crucial anatomical relationships with adjacent vessels that lead to an accurate and fluent procedure. Furthermore, the shortcomings of CT and/or MRI images, which are used as a guide for conventional hepatectomy, can be overcome with more intuitive and multidirectional anatomical information provided by the MI-3DVS. Therefore, the incidence of postoperative complications could be minimized with more parenchyma reservation, less hepatic blood occlusion, and shorter operative duration.

After recurrence was diagnosed, although suitable treatments such as RFA, TACE, second hepatectomy, PEI, and sorafenib were suggested, more than 20% of patients in each group rejected additional intervention. The 5-year OS and RFS were 61.1% and 40.2% in the SR group and 39.5% and 22.3% in the RFA group, respectively. It has been reported that the 5-year OS was 60–80% in patients who underwent liver resection [26–28] and 40–70% in those who received RFA [28, 29]. The results of OS in patients who underwent MI-3DVS-guided SR in the present study were consistent with these randomized prospective trials on conventional liver resection. HCC disseminates through portal and hepatic veins and spreads in the same liver segments [30, 31]. Therefore, anatomical hepatectomy has been widely accepted by surgeons because safe resection margins for HCC can be achieved (theoretically, 1-2 cm outside the tumor margin), eliminating both primary lesions and microdisseminations simultaneously [32]. A prospective study with a larger sample size will be performed to compare the benefits of MI-3DVS-guided hepatectomy and conventional resection. For RFA, repeat insertions and ablations are needed for larger tumors. Secondly, the procedure depends greatly on the guidance of 2-dimensional ultrasonography to obtain an ideal ablative area in a 3-dimensional level. Furthermore, the invasiveness and proliferation ability of the tumor cells at the periphery may be accelerated if RFA is incomplete [33]. Thus, the advantage of MI-3DVS-guided liver resection over RFA for small HCC could be the result of a more successful eradication.

The RFS of the RFA group in the present study was similar to that reported in previous clinical trials [26, 27] and lower than that reported in two larger sample size and multicenter retrospective studies. This disadvantage may have been caused by the higher number of patients with multifocal HCC (34/102 versus 183/1305) [34] and those with serum AFP ≥ 400 *μ*g/L (42/102 versus 34/319) [35] in the present study. Additionally, the poor access to adequate treatment facilities caused by the lower income level than that of developed countries could also be a reason for this difference to some extent [36].

As multiple lesions exist in cases of solitary HCC ≤ 3 cm only according to the Milan criteria, we divided the patients into three subgroups in which both tumor number and size were considered (solitary HCC ≤ 3 cm, solitary HCC > 3 cm and ≤5 cm, and multiple lesions) when survival analysis was performed rather than dividing the patients according to tumor number or diameter only. At the same time, this grouping method was adequate considering the superiority of RFA in ablating lesions no more than 3 cm in diameter [37]. The results of survival analysis between subgroups demonstrated that patients benefit more from hepatectomy than from RFA except for OS in older patients (aged > 60 years) and RFS in patients with multiple lesions and Child-Pugh class B and in older patients (aged > 60 years). Thus, RFA may be more suitable for older patients [29].

Factors associated with OS in bilateral correlation analysis were intervention, tumor number, tumor diameter, serum AFP, liver cirrhosis, Child-Pugh class, and tumor recurrence. Corresponding parameters associated with RFS were intervention, tumor number, tumor diameter, serum AFP, and Child-Pugh class. Recently, a study suggested that hepatitis virus was an independent prognostic factor in HCC patients [34]. Hence, we included hepatitis virus infection as a potential factor associated with prognosis when Cox regression analyses were performed, although there was no significant correlation between hepatitis and survival in the correlation analysis. The final Cox hazards model of our study demonstrated that independent predictive parameters for both OS and RFS were intervention, tumor number, and serum AFP. Resent publications indicated that older age and liver cirrhosis were risk factors associated with OS [34, 38, 39]. This difference could have been caused by the relatively small sample size as well as the epidemiologic characteristics in the current study.

The present study has some limitations. First, the presents study is limited by the retrospective study design, and the significance of the findings is not as strong as that provided by prospective studies or other study designs [40, 41]. Second, some patients received additional therapies such as RFA, TACE, and sorafenib because of tumor recurrence after initial treatment during the follow-up period. Thus, the OS may be cofounded to some extent by the availability of adequate medical services, although there was no significant difference between the two groups, especially for the subjects with lower income who tend to request RFA. Third, the comparison of long-term outcomes of MI-3DVS-guided hepatectomy and conventional liver resection was not assessed in the present study because a larger sample size was needed. Finally, some commonly accepted parameters associated with poor survival, such as histological differentiation and tumor staging, were not analyzed because not enough data were available in the RFA group.

## 5. Conclusion

MI-3DVS-guided hepatectomy should be considered as the primary treatment for HCC patients with multifocal disease, higher AFP level, and preserved liver function within the Milan criteria. However, for older candidates, RFA can be considered as an alternative therapy, as it could lead to comparable survival but shorter hospital stay and lower incidence of complications. Intervention, tumor number, and serum AFP are important and independent prognostic predictors of both survival and recurrence.

## Figures and Tables

**Figure 1:** Representative visualization results of small hepatocellular carcinoma and its spatial relationship with surrounding structures. (a) Overall location of the lesion; (b, c, d) the relationship between the tumor and hepatic vein (b), portal vein (c), and artery (d).

**Figure 2:** Overall survival and recurrence-free survival in the two groups. The 5-year overall survival rates were 61.1% and 39.5% in the SR and RFA groups, respectively. The 5-year recurrence-free survival rates were 40.2% and 22.3% in the SR and RFA groups, respectively. Both overall survival (*p* < 0.001) and recurrence-free survival (*p* = 0.002) were significantly higher in the SR group than in the RFA group. SR, three-dimensional visualization system-guided surgical resection; RFA, radiofrequency ablation.

**Table 1:** Clinical and demographic characteristics of patients in the two groups.

Variables	Group		Chi-square	*p *value
	SR (*n*)	RFA (*n*)		
Number of cases	92	102		
Gender (male/female)	75/17	90/12	*χ* ^2^ = 1.715	0.190
Age (years)	52.48 ± 8.36	54.02 ± 7.66	*t* = −1.340	0.182
Cases (age ≤ 60/>60)	77/15	8220	*χ* ^2^ = 0.357	0.550
Hepatitis			*χ* ^2^ = 1.712	0.634
None	12	17		
HBV	67	73		
HCV	6	8		
Both HBV and HCV	7	4		
Cirrhosis	49	49	*χ* ^2^ = 0.528	0.468
Alcoholism	13	7	*χ* ^2^ = 2.763	0.096
Diameter (cm)	3.19 ± 0.98	3.10 ± 0.88	*t* = 0.600	0.549
Tumor number (1/2/3)	67/18/7	67/22/13	*χ* ^2^ = 1.689	0.430
ALT (*μ*/L)	47.05 ± 28.55	43.32 ± 28.35	*t* = 0.912	0.363
AST (*μ*/L)	43.70 ± 28.05	49.15 ± 26.65	*t* = −1.388	0.167
Tbil (*μ*mol/L)	14.27 ± 7.44	16.52 ± 9.60	*t* = −1.809	0.072
ALB (g/L)	38.00 ± 4.75	39.36 ± 4.81	*t* = −1.969	0.050
Hb (g/L)	130.09 ± 17.39	132.63 ± 26.28	*t* = −0.806	0.422
PLT (≥10^11^/L/<10^11^/L)	84/8	89/13	*χ* ^2^ = 0.822	0.365
PT (≥15 sec/<15 sec)	20/96	11/83	*χ* ^2^ = 1.266	0.260
AFP (<400 *μ*g/L/≥400 *μ*g/L)	50/42	60/42	*χ* ^2^ = 0.395	0.530
Child-Pugh (A/B)	79/13	83/19	*χ* ^2^ = 0.565	0.452
Hospital stays (days)	18.04 ± 7.11	13.06 ± 5.59	*t* = 5.455	<0.001

HBV: hepatitis B virus; HCV: hepatitis B virus; ALT: alanine aminotransferase; AST: aspartate aminotransferase; Tbil: total bilirubin; ALB: albumin; Hb: hemoglobin; PLT: platelet; PT: prothrombin time; AFP: *α*-fetoprotein.

**Table 2:** Postoperative complications in the two groups.

Complication & classification	Group		Chi-square	*p* value
	SR (*n*)	RFA (*n*)		
Complications (totle)	38	20	*χ* ^2^ = 10.864	0.001
Hydrothorax	4	2		
Ascites	7	2		
Bile leakage	2	—		
Postoperative hemorrhage	1	1		
Hepatic failure	—	1		
Massive necrosis	—	1		
Pneumothorax	—	3		
Febrile (>38.5°C & >3 days)	5	2		
Pain (PCA included)	23	8		
Clavien-Dindo Classification			*z* = −2.094	0.036^*∗*^
Grade 1	19	16		
Grade 2	16	3		
Grade 3-4	3	1		

^*∗*^Mann-Whitney *U* test;

PCA: patient controlled analgesia.

**Table 3:** Treatments for tumor recurrence.

	Group		
Treatments	SR (*n* = 52)	RFA (*n* = 72)	*p* value
Without intervention	12	16	0.911
TACE	18	17	0.179
RFA	9	20	0.174
PEI	2	4	>0.999^*∗*^
Sorafenib	3	5	>0.999^*∗*^
Second hepatectomy	5	2	0.129^*∗*^
TACE and RFA	3	8	0.302

^*∗*^Fisher's exact test.

**Table 4:** Overall survival and recurrence-free survival for patients in subgroups.

Subgroups	5-year overall survival rate			5-year recurrence-free survival		
	SR (*n*)	RFA (*n*)	*p* value	SR	RFA	*p* value
Solitary > 3 cm	51.0% (39)	38.4% (44)	0.031	43.2%	26.7%	0.037
Multiple tumors	38.8% (25)	17.6% (34)	0.024	10.6%	7.0%	0.164
Solitary ≤ 3 cm	92.6% (28)	70.2% (24)	0.026	64.3%	36.2%	0.007
AFP < 400 *μ*g/L	73.6% (50)	47.8% (60)	0.002	50.9%	27.6%	0.002
AFP ≥ 400 *μ*g/L	46.9% (42)	28.5% (42)	0.008	26.8%	14.4%	0.027
Noncirrhosis	67.7% (43)	46.0% (53)	0.006	45.4%	25.5%	0.005
Cirrhosis	55.4% (49)	31.5% (49)	0.005	35.5%	17.9%	0.013
Child-Pugh A	64.8% (69)	45.2% (73)	0.002	42.3%	25.5%	0.002
Child-Pugh B	49.9% (23)	22.8% (29)	0.034	33.6%	11.9%	0.089
Age ≤ 60 years	63.2% (77)	36.8% (82)	<0.001	41.2%	22.2%	<0.001
Age > 60 years	60.0% (15)	51.0% (20)	0.814	35.6%	22.9%	0.709

AFP: *α*-fetoprotein.

**Table 5:** Correlation analysis of variables relevant to overall survival and recurrence-free survival.

	Overall survival (months)		Recurrence-free survival (months)	
Variable	Related coefficient	*p* value	Related coefficient	*p* value
Intervention^*∗*^	−0.325	<0.001^△^	−0.312	<0.001^△^
Gender^*∗*^	−0.024	0.735	0.002	0.981
Tumor number^$^	−0.590	<0.001	−6.16	<0.001
PLT^*∗*^	−0.056	0.437	−0.076	0.290
PT^*∗*^	−0.031	0.671	−0.005	0.941
Hepatitis^*∗*^	0.005	0.945	−0.009	0.900
AFP^*∗*^	−0.165	0.022^⋄^	−0.209	0.004^△^
Cirrhosis^*∗*^	−0.179	0.012^⋄^	−0.123	0.087
Child-Pugh class^*∗*^	−0.206	0.004^△^	−0.164	0.023^⋄^
Alcoholism^*∗*^	0.050	0.489	−0.008	0.908
Tumor diameter^$^	−0.381	<0.001	−0.340	<0.001
Tumor recurrence	−0.234	0.001^△^	—	—
Age (years)^#^	−0.096	0.185	−0.059	0.414
ALT (*μ*/L)^#^	0.078	0.280	0.087	0.226
AST (*μ*/L)^#^	0.037	0.612	0.059	0.441
Tbi (*μ*mol/L)^#^	0.074	0.305	0.047	0.513
ALB (g/L)^#^	0.072	0.321	0.047	0.517
Hb (g/L)^#^	0.042	0.559	0.004	0.957

^*∗*^Spearman correlation coefficient; ^#^Pearson correlation coefficient; ^$^partial correlations: diameters/tumor number were controlled while tumor number/diameters were analyzed. ^Δ^Correlation is significant at the 0.01 level (2-tailed). ^⋄^Correlation is significant at the 0.01 level (2-tailed). PLT: platelet; PT: prothrombin time; AFP: *α*-fetoprotein; ALT: alanine aminotransferase; AST: aspartate aminotransferase; Tbil: total bilirubin; ALB: albumin; Hb: hemoglobin.

**Table 6:** Univariate and multivariate analyses for overall survival.

Variables	Univariate analysis		Multivariate analysis	
	Score	*p *value	HR (95% CI)	*p* value
Survival				
Intervention (RFA versus SR)	14.118	<0.001	2.769 (1.789–4.286)	<0.001
Hepatitis virus infection	6.798	0.079		
HBV	6.598	0.010		
HCV	2.421	0.120		
Both HBV and HCV	0.531	0.466		
Liver cirrhosis	1.968	0.161		
Diameter (cm)	2.947	0.086	2.166 (1.656–2.835)	<0.001
Tumor number	61.910	<0.001	5.128 (3.548–7.413)	<0.001
AFP (≥400 *μ*g/L versus <400 *μ*g/L)	10.157	0.001	1.871 (1.229–2.847)	0.003
Child-Pugh (B versus A)	5.201	0.023		

HR: hazard ratio; SR: three-divisional visualization system-guided surgical resection; RFA: radiofrequency ablation; HBV: hepatitis B virus; HCV: hepatitis B virus; AFP: *α*-fetoprotein.

**Table 7:** Univariate and multivariate analyses for recurrence-free survival.

Variables	Univariate analysis		Multivariate analysis	
	Score	*p *value	HR (95% CI)	*p* value
Intervention (RFA versus SR)	12.264	<0.001	1.933 (1.340–1.789)	<0.001
Hepatitis virus infection	5.802	0.122		
HBV	3.523	0.061		
HCV	3.728	0.053		
Both HBV and HCV	0.284	0.594		
Liver cirrhosis	1.586	0.208		
Diameter (cm)	0.066	0.798	1.411 (1.132–1.759)	0.002
Tumor number	78.531	<0.001	3.903 (2.819–5.404)	<0.001
AFP (≥400 *μ*g/L versus <400 *μ*g/L)	7.146	0.008	1.474 (1.023–2.126)	0.038
Child-Pugh (B versus A)	3.865	0.049		

HR: hazard ratio; SR: three-divisional visualization system-guided surgical resection; RFA: radiofrequency ablation; HBV: hepatitis B virus; HCV: hepatitis B virus; AFP: *α*-fetoprotein.
